# Combined rs‐fMRI study on brain functional imaging and mechanism of RAGE‐DAMPs of depression: Evidence from MDD patients to chronic stress‐induced depression models in cynomolgus monkeys and mice

**DOI:** 10.1002/ctm2.541

**Published:** 2021-10-12

**Authors:** Weixin Yan, Lingpeng Xie, Yanmeng Bi, Ting Zeng, Di Zhao, Yuqi Lai, Tingting Gao, Xuegang Sun, Yafei Shi, Zhaoyang Dong, Ge Wen, Lei Gao, Zhiping Lv

**Affiliations:** ^1^ School of Traditional Chinese Medicine Southern Medical University Guangzhou Guangdong China; ^2^ The First Affiliated Hospital of Guangzhou University of Chinese Medicine Guangzhou Guangdong China; ^3^ College of Integrated Traditional Chinese and Western Medicine Jining Medical University Jining Shandong China; ^4^ Department of General practice The First Affiliated Hospital/School of Clinical Medicine of Guangdong Pharmaceutical University Guangzhou Guangdong China; ^5^ School of Fundamental Medical Science Guangzhou University of Chinese Medicine Guangzhou Guangdong China; ^6^ School of Nursing, Guangzhou University of Chinese Medicine Guangzhou Guangdong China; ^7^ Department of Medical Imaging Nanfang Hospital Southern Medical University Guangzhou Guangdong China; ^8^ Zhujiang Hospital Southern Medical University Guangzhou Guangdong China

**Keywords:** chronic stress, depression, functional connectivity (FC), prefrontal cortex (PFC), receptor for advanced glycation end products (RAGE), regional homogeneity (ReHo), resting‐state magnetic resonance imaging (rs‐fMRI)

## Abstract

More and more evidence show that major depressive disorder (MDD) is closely related to inflammation caused by chronic stress, which seriously affects human physical and mental health. However, the inflammatory mechanism of depression and its effect on brain function have not been clarified. Based on resting‐state functional magnetic resonance imaging (rs‐fMRI), we investigated change of brain functional imaging and the inflammatory mechanism of damage‐related molecular patterns (DAMPs)—receptor of advanced glycation protein end product (RAGE) in MDD patients and depressive‐like cynomolgus monkeys and mice models induced by chronic stress. The regional homogeneity (ReHo) and functional connectivity (FC) were analyzed using MATLAB and SPM12 software. We detected the expression of DAMPs‐RAGE pathway‐related proteins and mRNA in MDD peripheral blood and in serum and brain tissue of cynomolgus monkeys and mice. Meanwhile, RAGE gene knockout mice, RAGE inhibitor, and overexpression of AVV9^RAGE^ adeno‐associated virus were used to verify that RAGE is a reliable potential biomarker of depression. The results showed that the ReHo value of prefrontal cortex (PFC) in MDD patients and depressive‐like cynomolgus monkeys was decreased. Then, the PFC was used as a seed point, the FC of ipsilateral and contralateral PFC were weakened in depressive‐like mice. At the same time, qPCR showed that RAGE and HMGB1 mRNA were upregulated and S100β mRNA was downregulated. The expression of RAGE‐related inflammatory protein in PFC of depressive‐like monkeys and mice were consistent with that in peripheral blood of MDD patients. Moreover, the results were confirmed in RAGE*^–/–^* mice, injection of FPS‐ZM1, and overexpression of AAV9^*RAGE*^ in mice. To sum up, our findings enhance the evidence that chronic stress‐PFC‐RAGE are associated with depression. These results attempt to establish the links between brain functional imaging, and molecular targets among different species will help to reveal the pathophysiological mechanism of depression from multiple perspectives.

## Graphical abstract

1. The regional homogeneity value in prefrontal cortex (PFC) of MDD patients and depressive‐like monkeys were decreased and related to the upregulation of RAGE in peripheral or PFC.
2. RAGE is essential for the susceptibility of chronic stress to depression via regulating the functional connectivity of PFC in mice.
3. Overexpression or knockout/inhibition of RAGE in PFC can regulate depressive‐like behavior in mice.

## 1 INTRODUCTION

Major depressive disorder (MDD) is considered to be a complex and recurrent heterogeneous disease characterized by persistent and severe depression, decreased interest, accompanied by insomnia and hopelessness. WHO pointed out that depression has become the world's second largest disease and a major factor in the global burden of disease.^1^, ^2^, ^3^, ^4^ More and more evidence show that depression is closely related to chronic stress and immune inflammation activation.^5^, ^6^, ^7^ Brain‐derived neurotrophic factor (BDNF) and neurotransmitter 5‐hydroxytryptamine (5‐HT) are widely distributed in the key areas of the neural circuit and participate in the regulation of depression. The increase of proinflammatory cytokines/chemokines is directly involved in the pathophysiological process of stress‐related mental disorders (especially MDD), such as IL‐17A, IL‐1β, TNF‐α, etc.^7^, ^8^ and lead to the decrease of BDNF and 5‐HT levels. Therefore, the activation of immune inflammation mediated by chronic stress is of great significance to explore brain function regulation mechanism of MDD patients and depressive‐like animal models.

As a fast, noninvasive and radiation‐free image detection technology, fMRI has been widely used in neuroscience, pharmacology, and psychiatry. Research shows that there are many interrupted network connectivity in MDD core network, such as default mode network, and the limbic system and so on.^9^, ^10^ The analysis of functional connectivity (FC) is based on seed points and relies on a priori hypothesis. The changes of voxel activity over time (such as regional homogeneity [ReHo] and low‐frequency fluctuation amplitude [ALFF]) can help to reveal the changes of cerebral blood flow in patients with stress‐induced MDD.^11^ It is well known that ReHo is an important indicator of local nerve connectivity, which can more sensitively describe regional dysfunction and explain the dynamic characteristics of the time course of adjacent voxels.^12^, ^13^ It has been found that the increase of inflammation can cause the lack of pleasure, the decrease of ReHo, and the damage of brain network integrity in patients with depression.^14^ Moreover, the severity of depression also had a significant effect on ReHo. When HAMD score was high, ReHo in PFC (right middle frontal gyrus) decreased.^13^ It is worth noting that the PFC is the most closely related to human emotional psychology. It is not only related to many high‐level cognitive functional brain areas but also has extensive neural projections in other cerebral cortex and subcortical structures. Therefore, the relationship between chronic stress‐induced MDD patients and animal models with depressive‐like behavior and the study of specific brain regions can better reveal the mechanism of depression.

Stress is the main risk factor of depression. Under repeated or severe exposure to stressors, it can promote the occurrence of neuroinflammation through the release of damage‐related molecular patterns (DAMPs), and then affect the emotional and mental health. At present, the known DAMPs include high‐mobility group protein 1 (HMGB1), adenosine triphosphate, S100 protein, and others. Pattern recognition receptors (PRRs), such as receptor for advanced glycation end products (RAGE) and toll like receptors (TLRs), are recognized and connected on the cell surface to further activate the assembly and initiation of inflammasome.^15^, ^16^ RAGE exists on the cell membrane and is the key multiligand receptor for the expression and signal transduction of DAMPs and is also the core of signal transduction leading to chronic inflammation. Studies have found that RAGE can induce neuronal stress injury and microglia activation, participate in oxidative stress, immune activation, aging, and so on.^15^, ^16^ RAGE deletion mutant mice were resistant to chronic unpredictable stress‐induced behavior defects. The continuous increase of RAGE in microglia contributes to the initiation of depressive‐like behavior induced by chronic stress.^16^ Moreover, the RAGE/CREB‐NF‐κB signaling pathway in hippocampal DG is involved in the regulation of GLT‐1 expression, which may be related to chronic stress.^17^ Although preclinical and clinical evidence suggests that inflammation‐dependent DAMPs‐RAGE signaling can lead to emotional disorders, the effects of this signal on brain function and behavior of MDD patients and animals with depressive‐like behavior need to be further explored.

Therefore, we boldly hypothesized that the pathogenesis of depression is that chronic stress and other factors can activate the inflammatory‐related molecular pathways, further affecting the activity of brain regions and resulting in the occurrence of depression and depressive‐like behavior. We studied the mechanism of rs‐fMRI and DAMPs‐RAGE in MDD patients, nonhuman primate and rodent models of depression, and combined with RAGE knockout mice, RAGE inhibitor (FPS‐ZM1), and AAV9*^RAGE^* overexpression to further verify the molecular mechanism of RAGE in depression and its effect on behaviors.

## 2 METHODS AND MATERIALS

### 2.1 Subjects and ethical statement

#### 2.1.1 Human participants

All the subjects were from Guangdong 999 Brain Hospital and they were right‐handed Han, aged from 18 to 52 years old. The eligible participants enrolled in this study were (1) adults who matched the DSM‐IV diagnostic criteria and (2) the 24‐item Hamilton Scale for Depression (HAMD) to the single episode and severity of MDD. MDD patients with HAMD score ⩾ 17 were finally enrolled in this study. (3) No psychotropic drugs including antidepressants, benzodiazepines, sedative hypnotics, and mood stabilizers were taken within 2 weeks before MRI scanning and blood samples collection. In addition, MDD participants with mental history, other mental disorders, and illegal drug use were excluded. Healthy control participants were recruited from the physical examination center, (1) did not match the diagnostic criteria for MDD; (2) did not take any drugs for at least 4 weeks prior to the research; and (3) had no family history of mental and other systemic diseases.

This research had been registered on Chinese Clinical Trial Registry (http://www.chictr.org.cn, No. ChiCTRIPR‐14005427). All enrolled participants were informed of the research procedures and signed written informed consents. It was approved by Ethics Committee of Guangzhou Psychiatric Hospital. All procedures are fit to the Code of Ethics of the World Medical Association. Finally, 46 MDD patients and 54 healthy controls were recruited into this study. Data of participants were collected, such as gender, age, body mass index (BMI), and course of disease. Blood samples were collected from each subject before or within 24 h after MR scan.

#### 2.1.2 Nonhuman primates—monkeys

Fifteen healthy adult male (aged 6–7 years) cynomolgus monkeys were purchased from Blooming‐Spring Biological Technology Development Co., Ltd (Guangdong, China). The site of the study located at the Nanfang Hospital‐Experimental Animal Research Center, Guangzhou, China. Monkeys were randomly divided into three groups: a 12‐week social plus visual isolation‐induced depressive‐like cynomolgus group (SVC [12w], *n* = 5), SVC(16w) group experienced 12 weeks of social plus visual isolation with 4 weeks of recovery (*n* = 5), and a nonisolated control group (CON, *n* = 5). The rs‐fMRI data of monkeys were collected at 0th, 12th, and 16th weeks.

All experimental procedures of monkeys were conducted in strict accordance with the National Institutes of Health Guidelines (NIH Publication No. 8023, revised in 1978) and the Guide for the Care and Use of Laboratory animals for animal research and were approved by the Ethics Committee of Nanfang Hospital (Permit Number: NFYY‐2014‐53).

#### 2.1.3 Mice

Male 6‐ to 8‐week‐old C57BL/6J mice were purchased from Guangzhou Qingle Life Science Co., Ltd. (China), and male RAGE knockout mice (C57BL/6J background) aged 6–8 weeks were obtained from Professor Qiaobing Huang, School of basic medicine, Southern Medical University. The *RAGE^–/–^* mice identification is noted in Figure S4. In the experiment of brain function mechanism in mice (Figure 4A, F), the mice were randomly divided into the following groups: Control group, chronic unpredictable mild stress (CUMS) group, Control*^RAGE–/–^* group, and CUMS*^RAGE–/–^* group, *n* = 8/group. Among them, CUMS and CUMS *^RAGE–/–^* groups were given CUMS program for 6 weeks.^18^ After behavioral experiment, rs‐fMRI of anesthetized mice in each group was scanned (see Rs‐fMRI data acquisition for mice for details). In the experiment of FPS‐ZM1 administration (Figure 6A), animals were randomly divided into vehicle group, the CUMS+vehicle group, FPS‐ZM1 group, and CUMS+FPS‐ZM1 group, *n* = 8/group. The vehicle mice and CUMS mice were intraperitoneally injected with saline. FPS‐ZM1 group and CUMS+FPS‐ZM1 mice were intraperitoneally injected with FPS‐ZM1 ( 3  mg/kg/d, 6 weeks),^19^ and the mice in CUMS group and CUMS+FPS‐ZM1 group were established by CUMS program for 6 weeks at the same time. In the RAGE overexpression experiment (Figure 6K), animals were randomly divided into AAV9*^RAGE^* group and AAV9*^hSyn‐GFP^* group, *n* = 8–12 /group. AAV9*^RAGE^*/AAV9*^hSyn‐GFP^* (0.5 μl on each side) was injected into the PFC of mice by stereotactic injection (see Supplementary Material for details), and the scalp was sutured and fed for 3 weeks. Behavioral tests were performed before sacrificed. The principle of all mice experiments were the same as that of monkey experiments and were approved by the Ethics Committee of Nanfang Hospital (License No.: NFYY‐2014‐53).

### 2.2 SVC procedure for monkeys

Before this study, all monkeys grew up together in a stable social colony. Each monkey in the three groups was separately transferred to a standard size cage (1.6 × 1.2 × 1.2 m^3^), which located in a quiet room for 2 weeks of environmental adaptation and behavior observation. After that, five con monkeys returned to the large cage colony, were free to get food and water, and were raised under light/dark cycle for 12/12 h. The monkeys in SVC (12w) and SVC (16w) groups were transferred to modified small cages (0.4 × 0.3 × 0.5 m^3^), with four blinds around them. Each monkey in the SVC group was placed in a separate room, unable to receive the sound and smell of their peers.^20^ The activity space of them was smaller, but it did not affect eating, water intake, and defecation. After the 12th weeks, all monkeys were moved back to the standard single cage for continuous observation of behavior for 1 week. Rs‐fMRI data and serum were collected and SVC (12w) monkeys were sacrificed to collect brain tissue samples. The rest of the monkeys were transferred back to the large cage colony until the 16th week when they were again separately transferred to the standard single cages for continuous observation of behaviors (see Figure S1). Rs‐fMRI data, serum, and brain tissue were collected. The design of the monkey experiment is shown in Figure 2A.

### 2.3 Behavior observation of cynomolgus monkeys

The behavioral data of monkeys from 8:00 am to 11:30 am were recorded in detail and clearly by 30 high‐resolution cameras (Hikvision, China). The key observation time was 10:00–10:30 a.m., during which personnel were restricted to enter to interfere with monkeys. Ethogram defined categories derived from a basic rhesus monkey (ALTMANN, 1962). The main categories included measures of locomotor behavior, environmental exploratory behavior, anxious behavior, and rest behavior et al. During the 30‐min observation period, all records were analyzed and scored blindly by 3 well‐trained technicians who reached a consensus on behavioral classification, and the reliability among them was maintained at 85%–100%. Technicians used the focus tracking observation method and counted them in seconds. Scored behaviors were grouped into six categories: locomotor behavior, depressive‐like behavior, exploratory behavior, rest behavior, anxious behavior, and maintenance behavior. The body posture of curling up, slumping or collapsing with open eyes, inactivity accompanied by lack of response to environmental stimuli participated by other animals, were defined as depressive‐like behavior.^20^, ^21^, ^22^, ^23^, ^24^, ^25^ Anxious behavior included self‐scratching, body shakes, and yawning.^26^, ^27^ The behaviors of investigating cage, such as sniffing wall or bars and searching were regarded as exploratory behavior. Locomotor behaviors consisted of walking, jumping, running, and circling. Urination, defecation, eyes and hands rubbing, nail‐biting, and self‐grooming were all necessary maintain behavior. Rest behavior was regarded as siting awakened for ≥5 s, which is different from depressive‐like behavior.^20^, ^24^, ^25^, ^28^

### 2.4 CUMS procedure and behavioral tests for mice

Briefly, the CUMS procedure^18^ contains nine different stressors as follows: (1) 24 h of water and food deprivation, (2) night illumination, (3) 17 h of 45° cage tilted, (4) 5 min of swimming in 4°C water, (5) exposure to moist bedding for 24 h, (6) 12 h of empty bottle exposure, (7) disturbed cage for 24 h, (8) stimulated foreign body for 24 h, and (9) restricted exercise for 4 h. The CUMS procedure was used in different experimental designs, as depicted in Figures 4A, F and 6A.

After modeling, all mice underwent behavioral tests, tail suspension test (TST), sucrose preference test (SPT), and force swimming test (FST).^29^, ^30^ These tests were conducted by 3 well‐trained observers who were blinded to the mice conditions (see Supplementary Material for details).

### 2.5 Rs‐fMRI data acquisition

#### 2.5.1 Rs‐fMRI for human

All MR images were obtained on a clinical 3.0T HDXT scanner (GE, USA) equipped with a quadrature head coil. The whole‐brain high‐resolution three‐dimensional T1‐weighted images (3D‐T1WIs) was collected for brain segmentation and normalization^31^ and parameters: time of echo (TE) = 3.8 ms, time of repetition (TR) = 8.2 ms, flip angle = 7°, field of view (FOV) = 256 × 256 mm^2^, bandwidth = 191 Hz, voxel size = 1.0 × 1.0 × 1.0 mm^3^. Data were obtained using an echo‐planar imaging sequence (EPI) parameters: TE = 30 ms, TR = 2000 ms, flip angle = 90°, FOV = 240 × 240 mm^2^, bandwidth = 4131 Hz, voxel size = 3.4 × 3.4 × 3.4 mm^3^, 33 axial slices, and total volumes = 240. In addition, all sequence scans were carried out on each subject who excludes any clinical brain abnormalities. The preprocessing and ReHo analysis of all acquired rs‐fMRI images were analyzed by SPM12 and MATLAB software. The detailed steps are shown in the Supplementary Material.

#### 2.5.2 Rs‐fMRI for monkey

Before rs‐fMRI scans, monkeys were given atropine sulfate (0.05 mg/kg) and Telazol (3–5 mg/kg) via intramuscular injection to induce anesthesia, then endotracheal intubation and isoflurane inhalation anesthesia for scanning. The vital signs of the monkeys were monitored before and after the scan. All MR images were acquired using a 3.0T HDXT scanner (GE, USA) equipped with 8‐channel animal head coil (Figure S3). Single‐shot EPI was adopted with 400 time points, TE = 30 ms, TR = 1500 ms, matrix = 64 × 64, voxel size = 1.5 × 1.5 × 2.0 mm, number of excitations (NEX) = 1, slice thickness/gap = 2.0 mm/0 mm, flip angle = 69°, scan time = 10 min, 5 s. Moreover, for spatial normalization of intersubject brain fMRI, 3D‐T1WIs were scanned as structural images using a 3D‐BRAVO sequence with TR/TE/TI = 8/3/450, matrix = 230 × 230, voxel size = 0.70 × 0.7 × 0.7 mm, slice thickness/gap = 0.70/0 mm, NEX = 2, flip angle = 8°, scan time = 12 min, 51 s. Image preprocessing and regional homogeneity (ReHo) of each brain was calculated based on previously established quantification method of brain activity using SPM12, MATLAB software, and REST toolbox (http://restfmri.net/) as previously decribed.^32^ The detailed steps are shown in the Supplementary Material.

#### 2.5.3 Rs‐fMRI for mice

After the behavioral tests of mice, 7.0T small animal Bruker scanner (70/16 PharmaScan, Germany) was used for localization scanning of MRI. The mice were anesthetized with gas isoflurane (0%–0.3% isoflurane, 0.04 mg/kg/h S.C. of dexmedetomidine, 0.2 mg/kg i.p. of pancuronium bromide). Magnetic field intensity is 7.0 T and equipped with different sizes of animal surface coil and body coil, which can meet the imaging needs of the mouse's head and body. The experimental animals were fixed on the animal bed to reduce head movement. The respiratory frequency and heart rate of the animals were monitored by physiological monitor during the experiment. Hot water circulation system was used to maintain the normal body temperature of the experimental animal. Operation and processing system: paravision 6.0. EPI sequence with parameters: protocol = ax‐T1w, matrix size = 192 × 128, resolution = 0.14 × 0.14 × 1.0 mm, slice thickness = 1.4 mm, slice gap = 0.05 mm, TE = 9.01 ms, TR = 603.94 ms, averages = 32, scan time = 5 min, 10 s, volume = 1, repetitions = 1. The preprocessing of image and the functional connection value (CC value) and power spectrum were further analyzed and calculated by SPM12 and MATLAB software (see Supplementary Material for details). The threshold range of voxel level is 0.25–1.

### 2.6 Samples collection

Human serum were collected in a yellow separation gel tube and centrifuged at 3000 rpm for 10 min at room temperature (RT). Human blood samples were collected in vacutainer tubes with anticoagulant and erythrocyte lysis buffer was added in the ratio of 1:3 for fully lysed. Centrifuged at 3000 rpm for 5 min at RT, the white precipitate (i.e., peripheral leukocytes) was taken and mixed with Trizol to extract total RNA for RT‐qPCR. Telazol (3–5 mg/kg) and atropine sulfonate (0.05 mg/kg) were injected intramuscularly into cynomolgus monkeys for blood collection and the serum and peripheral leukocytes were collected respectively (the method is the same as above). The monkeys were euthanized by intravenous injection of over dose pentobarbital sodium solution. The heart was perfused with iced normal saline, and the brain tissues were taken after craniotomy. The mice were were euthanized by intraperitoneal injection of over dose pentobarbital sodium solution. Blood sample was quickly collected from the heart to separate serum (as above), and the brain was obtained by heart perfusion with iced PBS. All brain tissues were immediately packed according to the brain atlas and frozen in liquid nitrogen. All the samples were transferred and stored at –80℃ until further detection.

### 2.7 Detection of protein

The levels of 5‐HT in human and monkey serum were detected by ultra‐performance liquid chromatography‐mass spectrometry/mass spectrometry (UPLC‐MS/MS), RAGE level in serum of human and monkey were detected by RAGE enzyme linked immunosorbent assay (ELISA) Kit, and BDNF level in the serum of monkey and mouse were detected by BDNF ELISA Kit. The expressions of TLR4, NF‐κ B, RAGE, HMGB1, and S100β in prefrontal cortex of monkey and mouse were detected by Western blot (WB) and quantified by ImageJ software. The expression of RAGE, HMGB1, and S100β in prefrontal cortex was detected by immunofluorescence (IF) staining. The images were taken by laser confocal microscopy and analyzed by ImageJ software. The detailed steps of the above detection methods are shown in the Supplementary Material.

### 2.8 Quantitative polymerase chain reaction (QPCR)

The mRNA levels of RAGE, HMGB1, and S100β in human peripheral leukocytes and the mRNA levels of RAGE in PFC of monkeys and mice were detected by qPCR. The RNA was purified by Trizol and detected the concentration and purity of it by NanoDrop 2000 (Thermo Fisher Scientific, USA). Five hundred nanogram of total RNA was reverse transcribed into cDNA by reverse transcription kit (k1622, Thermo Scientific, USA). Primers for RAGE, HMGB1, and S100β were designed at https://www.ncbi.nlm.nih.gov/tools/primer‐blast/ (Table S2), and qPCR was performed on the ABiosystems 7500 (USA) using SYBR Green (420A, Takara, Japan). Cycle threshold values were normalized to GAPDH.

### 2.9 Statistical analysis

Differences in age, height, weight, BMI, education, HAMD, and SDS score between MDD and CON groups were evaluated by the two‐sample *t*‐test, or Mann–Whitney *U* test for nonnormally distributed data by SPSS 21.0 software. All correlation analyses were performed using Spearman's correlation with a significance threshold of *p* = .05 (Bonferroni correction). Differences in gender was assessed using the *χ* ^2^ test. Experimental data were expressed as the means ± SEM. Two‐group comparisons were assessed with Student's *t*‐test. Multigroup comparisons were analyzed with one‐way ANOVA in combination with the Bonferroni's testing as post hoc test. All statistical analyses were carried out using GraphPad Prism 8.0.3 software. Repeated measurement variance analysis of mice body weight data. Statistical significance was assumed if *p* values <  .05.

## 3 RESULTS

### 3.1 Demographic and clinical characteristics

There was no significant difference in age, gender, BMI, brain size, education, head motion during MR scan between MDD and CON group. The scores of HAMD and SDS in MDD patients increased significantly (both *p*s < .001). See Table 1 for more details.

**TABLE 1:** Demographic and clinical characteristics of participates with MDD and healthy controls (CON)

Characteristic	MDD (*n* = 46)	CON (*n* = 54)	statistic	*p* Value
Gender (male/female)	21/25	23/31	*χ* ^2 ^= 0.094	.759
Age (years)	28 (19–44)	27 (18–52)	*Z *= –0.533	.596
Height (cm)	164.5 (149–177)	164 (154–178)	*Z* = –0.142	.887
Weight (kg)	58.67±1.083	59.83 ± 0.9999	*T *= 0.7865	.4335
BMI	21.69±0.3944	22.11 ± 0.3427	*T *= 0.8125	.4185
Right‐handed (%)	46 (100)	54 (100)	*—*	*—*
Duration of illness (months)	6 (1–51)	*—*	*—*	*—*
Education (years)	12 (9–18)	12 (9–16)	*Z* = –2.261	.087
HAMD score	28 (23–35)	2 (0–6)	*Z* = –8.619	<.001*
SDS score	75 (68–83)	25 (20–36)	*Z* = –8.599	<.001*

HAMD, Hamilton depression scale; SDS, Self‐Rating Depression Scale.

* Stands for having statistical significance; “mean ± SD” is applied for normally distributed data, and “median (range)” is used otherwise.

### 3.2 Changes of brain ReHo in MDD patients compared with CON

The activity of spontaneous neurons in the brain of patients with depression was investigated by rs‐fMRI. Compared with CON, the levels of ReHo in PFC, temporal cortex, insula, marginal cortex, occipital cortex, parietal cortex, and cerebellum decreased significantly (Figure 1A–C and Table 2). However, ReHo increased in partial temporal cortex, cerebellum, PFC, parietal cortex, and occipital cortex. The PFC plays a key role in the development of emotion. By analyzing the correlation between ReHo value of BA11 and BA9 area of the PFC and HAMD score, SDS score, we found that BA11 area and BA9 area were negatively correlated with HAMD scores (*r* = –0.319, *p* < .01; *r* = –0.3889, *p* < .001, Figure 1D, E), and BA11 area and BA9 area were also negatively correlated with SDS scores (*r* = –0.3418; *r* = –0.3987, both *ps* < .001, Figure 1F, G).

**FIGURE 1:** Study on the ReHo changes of brain rs‐fMRI and RAGE‐DAMPs in patients with MDD. (A)–(C) Compared with the normal subjects, images of the horizontal, coronal, and sagittal planes show the decrease of prefrontal cortex BOLD‐signal of rs‐fMRI in the MDD patients according to the results of the ReHo analysis. The correlation between the scores of HAMD depression scale and the brain ReHo values of BA11 region (D) and BA9 region (E) of prefrontal cortex, respectively. The correlation between the scores of SDS anxiety scale and the brain ReHo values of BA11 region (F) and BA9 region (G) of prefrontal cortex, respectively. (H) Levels of 5‐HT in serum of MDD patients and normal subjects. The correlation between the scores of HAMD (I), SDS (J) and levels of 5‐HT in serum, respectively. (K) Levels of RAGE in serum of MDD patients and normal subjects. The correlation between the scores of HAMD (L), SDS (M), and levels of RAGE in serum, respectively. Fold changes of RAGE (N), HMGB1 (O), S100β (P) mRNA expression in peripheral leukocytes of MDD patients and normal subjects. The correlation between the scores of HAMD and mRNA expression of RAGE (Q), HMGB1 (R), S100β (S) in peripheral leukocytes, respectively. The correlation between the scores of SDS and mRNA expression of RAGE (T), HMGB1 (U), S100β (V) in peripheral leukocytes, respectively. The data are presented as means ± SEM. Two sample *t*‐test, ^*^ *p* < .05, ^**^ *p* < .01, ^***^ *p* < .001, MDD patients versus normal subjects. Spearman's correlation was used with a significance threshold of *p* < .05. *n*  =  46, 54 (CON, MDD, respectively)

**TABLE 2:** Results of ReHo suppression between MDD patients with con

Brain regions	BA	Cluster size	Peak *T* value	Peak MNI coordinate		
				*X*	*Y*	*Z*
L. medial frontal gyrus	BA11	238	–4.2425	–6	57	–24
L. orbital gyrus						
L. medial frontal gyrus	BA9	59	–3.5505	–6	48	24
L. superior temporal gyrus	BA38	751	–4.3538	–36	18	–33
L. middle temporal gyrus						
Cerebelum_6_L	BA19	587	–4.2659	–45	–78	0
L. middle occipital gyrus	BA37					
L. fusiform gyrus						
Cerebelum_6_R	BA37	475	–4.2873	33	–60	–24
R. fusiform gyrus						
R. superior temporal gyrus	BA38	144	–3.8567	36	18	–21
R. inferior frontal gyrus	BA47					
R. superior temporal gyrus	BA22	741	–3.9183	63	–15	–3
R. precentral gyrus	BA13					
R. middle temporal gyrus	BA6					
R. lingual gyrus	BA18	79	–3.1644	12	–69	–6
L. cuneus	BA18	171	–3.3556	–9	–81	15
L. postcentral gyrus	BA3	149	–3.371	–42	–24	54
R. postcentral gyrus	BA3	107	–3.0709	42	–21	51
R. paracentral lobule	BA4	61	–3.0636	3	–39	66
L. postcentral gyrus	BA2	49	–3.2482	–21	–30	75

L., left; R., right; BA, Brodmann area; MNI, Montreal Neurological Institute.

*p *< .05, corrected by GRF method at voxel‐level *p *<  .001.

### 3.3 Expression of 5‐HT in serum of MDD patients

The level of 5‐HT in serum was detected by UPLC‐MS/MS; it was found that compared with CON group, MDD patients’ serum 5‐HT was decreased significantly (*p* < .001, Figure 1H). The level of 5‐HT in serum was negatively correlated with HAMD and SDS score (*r* = –0.6967; *r* = –0.6837, both *p*s < .001, Figure 1I, J).

### 3.4 Expression of inflammatory molecules in peripheral blood of MDD patients

The results of ELISA showed that compared with CON group, the serum RAGE concentration of MDD patients had an upward trend, but there was no statistical difference (*p* > .05, Figure 1K). No correlation was found between RAGE and HAMD score and SDS score (*r* = –0.09963, *r* = –0.07059, *p*s > .05, Figure 1L, M). QPCR results showed that compared with CON group, the fold change of RAGE and HMGB1 mRNA in peripheral blood nucleated cells of MDD patients were significantly increased (*p*s < .01, Figure 1N, O) and the fold change of S100β mRNA decreased (*p* < .05, Figure 1P). The the fold change of RAGE and HMGB1 mRNA were positively correlated with HAMD score (*r* = 0.2426, *p *< .05; *r* = 0.2399, *p *= .0505, Figure 1Q, R) and SDS score (*r* = 0.1824, *p *> .05; *r* = 0.2987, *p *< .05, Figure 1T, U). The fold change of S100β mRNA in peripheral blood nucleated cells was negatively correlated with HAMD score and SDS score (*r* = –0.2669, *r* = –0.2982, *p*s < .05, Figure 1S, V). There were no significant correlation between RAGE in serum and RAGE, HMGB1, S100β mRNA expression in peripheral blood nucleated cells and BA11 brain area (*r* = 0.2674, *p* < .05; *r* = 0.03905, *r* = –0.2154, *r* = –0.05096, *p*s > .05, see Figure S1A–D), The same trend was found in brain area of BA9 (*r* = 0.06358; *r* = 0.1092, *r* = –0.1929, *r* = 0.09816, *p*s > .05, see Figure S1E–H).

### 3.5 Behavioral and neurotransmitter changes in depressive‐like cynomolgus (SVC) induced by social plus visual isolation

The nonhuman primate model of depression was established as described previously, 10 male adult cynomolgus monkeys received 12 weeks of social plus visual isolation (Figure 2A). At the 12th week, the behavioral observation showed that compared with CON group, SVC (12W) monkeys showed depressive‐like behavior, crouching, head lower than shoulder, less activity, and less interest (see Figure S2). Among them, the total time and percentage of locomotor and exploratory behavior of SVC (12w) monkeys were reduced (*p *< .001; *p *< .05. Figure 2B, C), and the total time and percentage of depressive‐like and anxiety‐like behavior increased (both *ps* < .001. Figure 2D, E). There was no statistically significant difference in the total time and percentage of rest and maintain behavior (both *ps* > .05. Figure 2B, C). Simultaneously, the levels of BDNF and 5‐HT in serum of SVC (12w) monkeys were significantly lower than those in CON (both *p*s < .001, Figure 2D, E)

**FIGURE 2:** Social plus visual isolation establishes an effective depression model of cynomolgus monkeys and caused the ReHo changes of brain rs‐fMRI. (A) Schematic showing experimental approach and timeline. (B), (C) Quantification of total time and proportion of behavior time in different groups of cynomolgus monkeys. Levels of 5‐HT (D) and BDNF (E) in serum of cynomolgus monkeys. Compared with the CON group, images of the axial (F), coronal (G), and sagittal (H) planes show the BOLD‐signal changes of rs‐fMRI in the SVC group according to the results of the ReHo analysis at the 12th week. The data are presented as means ± SEM. One‐way ANOVA followed by Bonferroni's post hoc test, ^*^ *p* < .05, ^***^ *p* < .001. SVC (12w) group versus CON group; ^##^ *p* < .001, ^###^ *p* < .001. SVC (16w) group versus CON group; ^△^ *p* < .05. SVC (16w) group versus SVC (12w) group; *n*  =  5, 5, 5 (CON, SVC [12w], SVC [16w], respectively). The voxel‐level height threshold was *p *< .005 (uncorrected) and the cluster‐extent threshold was 20 voxels

### 3.6 The effect of social plus visual isolation on cynomolgus monkeys brain ReHo by rs‐fMRI

As shown in the axial (Figure 2F), coronal (Figure 2G) and sagittal (Figure 2H) planes, a series of fMRI signal changes based on blood oxygen level dependence, were induced by the social plus visual isolation exposure. ReHo analysis showed that at the 12th week, compared with the CON group, the main areas of brain with decreased ReHo value in SVC (12w) monkeys were the prefrontal cortex (area 8bs, 44T), premotor and motor cortex (area F3, F5_6Va_6Vb), somatosensory cortex (area 5_PE, 5_PEa), parietal cortex (area LIPd), visual cortex (area 7a_Opt_PG, 7b_PFG_PF), especially PFC. In contrast, the ReHo values of the PFC (area 8Ad, 8Av, 46d) and premotor and motor cortex (area F4) were increased, detailed in Table S1.

The ReHo values of SVC (12W) and SVC (16W) monkeys were compared by longitudinal analysis (see Figure 3A–C, Table S1). Compared with that at the 0th week, the areas of the brain with decreased ReHo value in SVC monkeys at the 12th week were as follows the PFC (area 10mr, 11m, 13a, 13b, 13m, 14c, 25t, 45a, 45b, 46d, 46v, 46f, 8Av), hippocampus (area CA3, CA4, DG, Sub, paraS), parahippocampal cortex (area TF, TH), striatum, premotor, and motor cortex (area F1_4, F5_6Va_6Vb, F2_6DR_6DC, F3), visual cortex (area V1). The ReHo values of the temporal cortex (area RTp, STGr), auditory cortex (area RT, RM), geniculate nucleus (area LGNp, Mgad, MGpd, MGv) were increased.

**FIGURE 3:** Social plus visual isolation exposure induced persistent decrease of ReHo value and increase of RAGE in PFC of cynomolgus monkeys. (A)–(C) The ReHo value changes of rs‐fMRI in PFC of SVC monkeys at different time points from three levels: horizontal, coronal and sagittal, respectively; (A) 12th week vs 0th week; (B) 16th week vs 0th week; (C) 16th week vs 12th week. The voxel‐level height threshold was *p *< .005 (uncorrected) and the cluster‐extent threshold was 20 voxels. (D) Expression of RAGE in serum of cynomolgus monkeys, *n*  =  5, 5, 5 (CON, SVC [12w], SVC [16w], respectively). (E) Relationship between RAGE expression in serum and depressive‐like behavior in cynomolgus monkeys. (F) Expression of RAGE mRNA in PFC of cynomolgus monkeys. (G), (H) Western blot and semiquantitative results of TLR4, NF‐κB, RAGE, HMGB1 and S100β in mPFC of cynomolgus monkeys. Relationship between 5‐HT (I) and BDNF (J) expression in serum and depressive‐like behavior in cynomolgus monkeys. (K) Relationship between the ratio of RAGE mRNA expression in PFC and depressive‐like behavior in cynomolgus monkeys. Immunofluorescence of HMGB1 (L), RAGE (M), and S100β (N) in mPFC of cynomolgus monkeys. White scale bar represents 10 μm. The data are presented as means ± SEM. One‐way ANOVA followed by Bonferroni's post hoc test. ^*^ *p* < .05, ^***^ *p* < .001. SVC (12w) group versus CON group; ^###^ *p* < .001. SVC (16w) group versus CON group; ^△△^ *p* < .01. SVC (16w) group versus SVC (12w) group. , Representative data from WB, qPCR, and IF at least 3 independent experiments are shown; *n*  =  5, 5, 5 (CON, SVC [12w], SVC [16w], respectively). Spearman's correlation was used with a significance threshold of *p* < .05

### 3.7 Behavior and brain ReHo of SVC (16w) cynomolgus monkeys at 4 weeks after modeling

In order to clarify the effects of chronic stress on the behavior, brain regions, and the stability of the model of cynomolgus monkeys, we also observed and evaluated the behavior and rs‐fMRI of SVC monkeys at the 16th week (Figure 2A). After 4 weeks of recovery, SVC (16w) monkeys still showed obvious depressive‐like behavior. The total time and percentage of locomotor behavior decreased significantly (*p *< .001. Figure 2B, C). The total time and percentage of depressive‐like and anxiety‐like behavior increased (both *ps* < .001. Figure 2B, C). There were no significant difference in exploratory, rest and maintain behavior (both *ps* > .05. Figure 2B, C). The level of BDNF and 5‐HT in SVC (16w) monkeys serum were increased (*p *< .01, *p *< .001, Figure 2D, E). However, compared with SVC (12w) monkeys, SVC (16w) monkeys still showed significantly depressive‐ike behavior, and there was no significant difference in total time and percentage (*p* > .05, Figure 2B, C). The total time and percentage of locomotory behavior increased (*p* < .001, Figure 2B, C), and the total time and percentage of anxiety‐like behavior and rest behavior decreased (*p* < .001; *p* < .05, Figure 2B, C). There was no significant difference in the total time and percentage of exploratory behavior and maintenance behavior (both *p* > .05, Figure 2B, C) and brain ReHo value. The levels of BDNF and 5‐HT in serum of SVC (16w) monkeys were increased (both *p*s < .05, Figure 2D, E).

Through the longitudinal analysis and comparison of SVC (16w) monkeys, it was found that at the 16th week compared with the 0th week, the areas with decreased ReHo were the PFC (area 12l, 13b, 13 m), amygdala (area Bi, Ld, Lv), hippocampal hippocampal (area CA3, DG), striatum, temporal cortex (area Ipa, Tga, Tead, Tem, Tepd, STGr, Taa, TPO, PGa), visual cortex (area V3v), and premotor and motor cortex (area F5_6Va_6Vb). The cerebellum was elevated in ReHo. Compared with the 12th week, cerebellum was decreased in ReHo, and the PFC (area 46d, 46v, 8bm, 9D) was increased in ReHo (Figure 3A–C, Table S1).

### 3.8 Increase of RAGE expression in in serum and PFC of SVC monkeys

The expression of RAGE in serum of cynomolgus monkeys was detected by ELISA. Compared with CON monkeys, the serum RAGE level of SVC (12w) cynomolgus monkeys increased (*p* < .05, Figure 3D). QPCR results showed that compared with CON monkeys, RAGE mRNA level in mPFC of SVC (12w) and SVC (16w) monkeys were significantly increased (*p* < .001; *p* < .01, Figure 3F). The expressions of TLR4, NF‐κB, RAGE, HMGB1, and S100β in mPFC of monkeys were detected by WB. The results indicated that the expressions of NF‐κB, RAGE, and HMGB1 were significantly increased (both *p*s < .001, Figure 3G, H) and S100β was significantly reduced (*p* < .05, Figure 3G, H). The expressions of HMGB1 and RAGE in mPFC of SVC (16w) were significantly increased (both *p*s < .001, Figure 3G, H). Meanwhile, compared with SVC (12w) monkeys, the expressions of NF‐κB and HMGB1 in mPFC of SVC (16w) monkeys were decreased (both *p*s < .01, Figure 3G, H). There were positive correlation between RAGE expression in serum and PFC and depressive‐like behavior in cynomolgus monkey (*r* = 0.6452, *p *< .01; *r* = 0.7758, *p *< .001, Figure 3E, K). Moreover, the IF results of RAGE, HMGB1, and S100β in the mPFC of SVC monkeys were consistent with of WB (Figure 3L–N). In addition, we found a negative correlation between the expression of 5‐HT and BDNF in serum and depressive‐like behavior of cynomolgus monkey (*r* = –0.97, *r* = –0.853, *ps *< .001, Figure 3I, J).

### 3.9 Decreased functional connectivity and increased RAGE expression in PFC of depressive‐like mice

In order to further study the mechanism of depression, we established a mouse CUMS depression model (Figure 4A). Behavioral tests showed that compared with control group, CUMS mice had significantly lower body weight (*p* < .001, Figure 4G), significantly reduced sucrose consumption (*p* < .001, Figure 4H), and longer immobility time of TST and FST (*p* < .001, Figure 4I, J), and the level of BDNF in serum was significantly induced by ELISA (*p* < .001, Figure 4K). The results of the interhemispheric or intrahemispheric functional connectivity of PFC showed that compared with control, the intensity of FC of the PrL and FrA in CUMS group was decreased and the area of connection was reduced (both *ps* < .001, Figure 5A–D). The FC between ipsilateral and contralateral hemispheres of PrL were decreased (both *p*s < .001, Figure 5E, G), and ipsilateral hemispheres of FrA was decreased (*p* < .05, Figure 5I). But there was no significant difference in the contralateral hemisphere (*p *> .05, Figure 5K). Meanwhile, qPCR results indicated that the fold change of RAGE mRNA in PFC of CUMS mice was increased (*p*s < .05, Figure 4B). WB results indicated that the protein expression of NF‐κB, RAGE, and HMGB1 in PFC of CUMS mice were increased (*p* < .01, *p* < .01, *p* < .05, Figure 4C, D), while the S100β was decreased (*p* < .001, Figure 4C, D). There was no significant difference in TLR4 expression (*p* > .05, Figure 4C, D). IF showed that RAGE expression in PFC of CUMS depressive‐like mice was significantly increased (Figure 4E).

**FIGURE 4:** RAGE knockout is resilient to CUMS Exposure and increase interhemispheric and intrahemispheric rs‐fMRI connectivity in PFC of mice. (A) Schematic overview of CUMS experimental approach and timeline. (B) The mRNA fold change of RAGE in PFC of mice were detected by qPCR. (C), (D) Western blot and semiquantitative results of TLR4, NF‐κB, RAGE, HMGB1 and S100β in PFC of mice. (E) Immunofluorescence expression of RAGE in PFC of mice. (F) Schematic showing experimental approach and timeline. The CUMS model was established in WT mice combined with RAGE*^–/–^* mice, and the brain was scanned with rs‐fMRI. (G) Body weight changes in mice, *n* = 8, respectively. Mice behavioral tests. (H) Sucrose preference test (SPT); (I) tail suspension test (TST); (J) force swimming test (FST), *n* = 8, respectively. (K) Expression of BDNF in serum of four groups of mice, *n* = 8, respectively. (L), (M) Western blot and semiquantitative results of TLR4, NF‐κB, RAGE, HMGB1, and S100β in PFC of mice. (N) Immunofluorescence showed that RAGE knockout could downregulate the expression of RAGE in PFC of CUMS depressive‐like mice. One‐way ANOVA followed by Bonferroni's post hoc test; ^*^ *p* < .05, ^**^ *p* < .01, and ^***^ *p* < .001, CUMS group versus Control group; ^#^ *p* < .05, ^##^ *p* < .01, and ^###^ *p* < .001, CUMS group versus CUMS*^RAGE–/–^* group; ^△^ *p* < .05, ^△△^ *p* < .01, and ^△△△^ *p* < .001, CUMS group versus Control*^RAGE–/–^* group; Error bars indicate mean ±SEM. White scale bar represents 10 μm. Representative data from WB, qPCR and IF at least 3 independent experiments are shown; *n*  =  8, 8, 8, 8 (Control, CUMS, Control*^RAGE–/–^*, CUMS*^RAGE–/–^*, respectively)

**FIGURE 5:** Effect of *RAGE* knockout on brain functional connectivity in depressive‐like mice induced by chronic stress. Rs‐fMRI connectivity maps of PrL in four groups of mice (A), corresponding quantification of interhemispheric connectivity (B). Rs‐fMRI connectivity maps of FrA in four groups of mice (C), corresponding quantification of interhemispheric connectivity (D). Quantification of intrahemispheric rs‐fMRI connectivity (E, G) and the respective power spectrum (F, H) of ipsilateral and contralateral PrL in four groups of mice. Quantification of intrahemispheric rs‐fMRI connectivity (I, K) and the respective power spectrum (J, L) of ipsilateral and contralateral FrA in four groups of mice. Rs‐fMRI maps generated by correlation analysis of band‐pass filtered (0.005–0.1 Hz) BOLD signals using a seed defined in the ipsilateral and contralateral side. Seed location is indicated by a blue crosshair. Quantification of the interhemispheric rs‐fMRI connectivity (*n* = 6). One‐way ANOVA followed by Bonferroni's post hoc test; ^*^ *p* < .05 and ^***^ *p* < .001, CUMS group versus Control group; ^#^ *p* < .05, ^###^ *p* < .001, CUMS group versus CUMS*^RAGE–/–^* group; ^△^ *p* < .05, ^△△△^ *p* < .001, CUMS group versus Control*^RAGE–/–^* group; Error bars indicate mean ± SEM

### 3.10 RAGE knockout can improve the behavior and brain functional connectivity of mice under chronic stress

We designed the experiment with RAGE*^–/–^* mice and collected rs‐fMRI data (Figure 4A). Statistical analysis revealed that there were no significant difference in power spectrum of the PrL and FrA of bilateral hemispheres between the groups (both *p*s > .05, Figure 5F, H, J, L). Then, compared with control, there were no obvious difference in body weight, behavioral test, serum BDNF level, protein expression of TLR4, NF‐κB, RAGE, HMGB1, S100β in PFC and functional connection of the PrL and FrA of Control*^RAGE–/–^* mice (both *p*s > .05, Figures 4G–N and 5A–E, G, I, K). Compared with CUMS group, CUMS*^RAGE–/–^* mice increased weight (*p *< .001, Figure 4G) and level of BDNF in serum (*p* < .001, Figure 4K), improved depressive‐like behavior, increased sugar water consumption, and reduced the immobility time of TST and FST (*p* < .001; *p* < .05; *p* < .001, Figure 4H–J). WB analysis reflected that the expressions of NF‐κB, RAGE, and HMGB1 were downregulated and S100β was upregulated in CUMS*^RAGE–/–^* mice (*p* < .01; *p* < .05; *p* < .01; *p* < .01; Figure 4L, M). IF showed that the expression of RAGE in PFC of CUMS*^RAGE–/–^* group was downregulated (Figure 4N).

At the same time, It was also found that compared with CUMS mice, rs‐fMRI connectivity and area between interhemispheres of the PrL and FrA in CUMS*^RAGE−/−^* mice were increased (*p *< .001; *p *< .05, Figure 5A–D). The FC of ipsilateral hemisphere of PrL increased in CUMS*^RAGE−/−^* mice (*p* < .05, Figure 5E). Although the FC in the contralateral of PrL and the bilateral of FrA hemispheres tended to increase, there was no statistical difference (both *ps* > .05, Figure 5G, I, K).

### 3.11 Inhibitor of RAGE (FPS‐ZM1) alleviated depressive‐like behavior induced by chronic stress and overexpression of AAV9^*RAGE*^ in PFC of mice increased the susceptibility to depression

Since the FPS‐ZM1 can pass through the blood–brain barrier, we intervened by intraperitoneal injection of FPS‐ZM1 in mice (Figure 6A). The results showed that compared with vehicle group, there are no significant difference in body weight, behavior test, serum BDNF level in PFC of FPS‐ZM1 group (both *p*s > .05, Figure 6B–H). Compared with CUMS+Vehicle group, CUMS+FPS‐ZM1 group significantly increased body weight (*p* < .05, Figure 6B) and serum BDNF level (*p* < .001, Figure 6C), increased sucrose consumption, and reduced the immobility time of TST and FST (both *ps* < .001, Figure 6D–F). WB result indicted that the expression of NF‐κB, RAGE, and HMGB1 significantly reduced in PFC of CUMS+FPS‐ZM1 group (*p* < .05; *p* < .001; *p* < .001; Figure 6G, H). IF showed that expression of RAGE lessened in PFC of CUMS+FPS‐ZM1 group (Figure 6I).

**FIGURE 6:** Inhibitor of RAGE(FPS‐ZM1) alleviated depressive‐like behaviors induced by CUMS and overexpression of AAV9*^RAGE^* in PFC increased the susceptibility to depression in mice. (A) Schematic showing experimental approach and timeline. Mice were intraperitoneally injected in FPS‐ZM1 or 0.9% saline for 6 weeks, once a day. FPS‐ZM1 can improve body weight (B) and the level of BDNF in serum of mice (C) after CUMS exposure, *n* = 8, respectively. FPS‐ZM1 alleviated depressive‐like behaviors induced by CUMS. (D) SPT; (E) FST; (F) TST, *n* = 8, respectively. (G), (H) Western blot and semiquantitative results of TLR4, NF‐κB, RAGE and HMGB1 in PFC of mice. (I) Immunofluorescence expression of RAGE in PFC of mice. (J) Experimental diagram of the overexpression of AAV9^hSyn‐GFP^/AAV9*^RAGE^* by stereotactic injected into the PFC of mice. (K) Relative mRNA levels of RAGE in the neurons of mice’ PFC transfected with AAV9*^hSyn‐GFP^* or AAV9*^RAGE^* are shown. (L) Representative images of AAV9*^hSyn‐GFP^*/AAV9*^RAGE^* viral infection in the medial PFC. White scale bar represents 10μm. Following 3‐week normal feeding and behavioral testing, the medial PFC was collected from a subset of mice for mRNA analyses. Mice infused with AAV9*^hSyn‐GFP^*/AAV9*^RAGE^* behavior tests. (M) SPT; (N) FST; (O) TST; *n* = 8, respectively. (P) Expression of BDNF in serum of mice after injection of AAV9*^hSyn‐GFP^*/AAV9*^RAGE^*, *n* = 8, respectively. (Q), (R) Western blot and semiquantitative results of NF‐κB and RAGE in PFC of mice after injection of AAV9*^hSyn‐GFP^*/AAV9*^RAGE^*. (S) Immunofluorescence expression of RAGE in PFC of mice after injection of AAV9*^hSyn‐GFP^* / AAV9*^RAGE^*. One‐way ANOVA followed by Bonferroni's post hoc test; ^**^ *p* < .01, ^***^ *p* < .001, CUMS+Vehicle group versus Vehicle group; ^#^ *p* < .05, ^##^ *p* < .01, and ^###^ *p* < .001, CUMS+FPS‐ZM1 group versus CUMS+Vehicle group; ^△△△^ *p* < .001, CUMS+Vehicle group versus FPS‐ZM1 group. Means significantly different from the AAV9*^hSyn‐GFP^* group and the AAV9 *^RAGE^* group based on two‐sample *t*‐test are denoted. ^▲▲^ *p* < .01, ^▲▲▲^ *p* < .001. Error bars indicate means ± SEM. White scale bar represents 10 μm. Representative data from WB, qPCR and IF at least 3 independent experiments are shown; *n*  =  8, 8, 8, 8, 8, 8 (Vehicle, CUMS+Vehicle, FPS‐ZM1, CUMS+FPS‐ZM1, AAV9*^hSyn‐GFP^*, AAV9*^RAGE^*, respectively)

To further confirm the key role of RAGE in PFC on depression. The behavioral changes of mice and the expression of DAMPs‐RAGE‐related proteins were observed after overexpression of AAV9*^RAGE^* adeno‐associated virus by stereotactic injected into PFC of mice (Figure 6J). Representative images of AAV9*^hSyn‐GFP^* or AAV9*^RAGE^* viral infection in PFC were shown in Figure 6L. The results of qPCR indicated that relative level of RAGE mRNA in PFC of AAV9*^RAGE^* group was significantly increased after 3 weeks of virus expression (*p < *.01, Figure 6K). The behavioral test showed that compared with AAV9*^hSyn‐GFP^* group, the sucrose preference of AAV9*^RAGE^* group was lower (*p < *.01, Figure 6M), and the immobility time of TST and FST was significantly longer (*ps < *.001, Figure 6N, O). The level of BDNF decreased in serum of AAV9*^RAGE^* group (*p < *.01, Figure 6P). We further confirmed the expression of inflammatory proteins by WB and found that the expression of NF‐κB and RAGE increased in PFC of AAV9*^RAGE^* group (*ps < *.001, Figure 6Q, R). IF also confirmed that RAGE was upregulated in PFC of AAV9*^RAGE^* group (Figure 6S). So we have reason to believe that the overexpression of RAGE in PFC of mice can increase the susceptibility to depression.

## 4 DISCUSSION

Previous depression studies have indicated that the activation of inflammatory molecules mediated by chronic stress is closely related to brain dysfunction. In this study, we used rs‐fMRI to investigate the brain imaging mechanism and DAMPs‐RAGE inflammatory mechanism of MDD patients and chronic stress‐induced depressive‐like cynomolgus and mouse models. In order to further study the target brain region, we analyzed the ReHo of human and monkey brain and the FC of mice. Combined with RAGE knockout mice, RAGE inhibitor (FPS‐ZM1) and overexpression of AAV9*^RAGE^* adeno‐associated virus verify the inflammatory protein markers of depression and its effect on behavior. At the same time, the inflammatory proteins in peripheral blood and brain were verified by Western blotting, qPCR, and ELISA. To sum up, our study shows that chronic stress can cause abnormal activation of emotion regulation‐related brain regions, upregulation of RAGE‐related inflammatory protein, and behavioral changes in MDD patients, depressive‐like cynomolgus, and mice. Furthermore, molecular imaging links between different species were established to better reveal the pathogenesis and treatment strategies of depression.

Previous studies on depression mainly focused on clinical MDD patients and rodent models. Due to ethical limitations, MDD and normal human brain tissue samples are difficult to obtain. Most of them can only indirectly reflect the pathogenesis of MDD from brain imaging and molecular detection. However, nonhuman primates are highly consistent with human in brain structure, cognitive function, behavior, and so on, and have obvious advantages in the study of depression. We can use the monkey depression model, the convenience of brain tissue, and brain imaging to supplement and verify the pathogenesis of clinical MDD. But due to the high price and large size of monkeys, rodent models can have more advantages in combination with targeted gene knockout, pathway inhibition, overexpression, and other ways to conduct in‐depth mechanism research. Therefore, chronic stress was used to establish depressive‐like cynomolgus and mouse models, and combined with clinical MDD patients to carry out molecular imaging research of depression. It is a practical, multifaceted, multilevel research combination and also the merits and highlights of this study. Studies have shown that social plus visual isolation can stably induce depressive‐like behavior in cynomolgus monkeys.^21^, ^22^, ^24^ Our study found that the curling behavior (head lower than shoulder) of SVC monkeys has been identified as the core behavior of depression in nonhuman primates.^22^, ^33^, ^34^ The total duration and proportion of locomotor behavior and exploratory behavior decreased, while the duration and proportion of depressive‐like behavior and anxiety‐like behavior increased. The levels of 5‐HT and BDNF in serum were decreased. These findings are consistent with previous studies on depression in cynomolgus monkeys. Interestingly, after 4 weeks of recovery, although the locomotor behavior increased and the anxiety‐like behavior decreased, SVC monkeys still showed obvious depressive‐like behavior. Moreover, the serum levels of 5‐HT and BDNF were still decreased, indicating that social plus visual isolation can maintain depressive‐like behavior of cynomolgus monkeys for at least 1 month, and the model was stable. At the same time, we established a 6‐week CUMS depression model in mice and found that the weight and serum BDNF of CUMS mice decreased, increased depressive‐like behavior, reduced the use of sucrose, and prolonged the immobility time of TST and FST, indicating that the mouse depression model was successfully established and laid a foundation for further research.

Rs‐fMRI is based on blood oxygen level to reflect the brain functional activity. ReHo reflects the consistency of local activity of brain neurons, is an important indicator of local nerve connectivity. Functional connectivity is a specific indicator of brain functional network connectivity based on the changes of specific brain areas. Previous studies have proved that the changes of ReHo mainly concentrated in prefrontal cortex in patients with MDD.^35^, ^36^ The PFC plays a key role in reward and emotion regulation network. The ReHo and FC of PFC have been considered to be major neurobiological basis related to the pathogenesis of MDD.^37^, ^38^ As we all know, serotonin (5‐HT) is a neurotransmitter, which is synthesized by tryptophan and regulated by emotion. It cannot pass directly through the blood–brain barrier unless with the help of ryptophan and transporters. The decrease of 5‐HT level in peripheral blood can indirectly reflect the level of 5‐HT, which may be closely related to indoleamine 2,3‐dioxygenase 1 (IDO1) and metabolism of tryptophan.^39^ Our results demonstrated that the level of 5‐HT in serum of MDD patients was significantly decreased, and the ReHo in BA11 and BA9 regions of PFC was decreased, which was consistent with the reported study.^40^ Second, we found that serum 5‐HT level and ReHo value of BA11 and BA9 were negatively correlated with HAMD and SDS score. At the same time, we also conducted the horizontal and longitudinal ReHo analysis of depressive‐like monkeys and found that the functional decline of PFC was consistent with the clinical MDD patients. After 4 weeks of recovery, ReHo increased in PFC of SVC monkeys, indicating that function of PFC was also recovering. In other words, we have reason to think that the reduction of PFC function may be an important mechanism of depression. However, the relationship between PFC dysfunction and brain functional connectivity is inseparable. As has been widely reported, ReHo is usually used to describe spontaneous cerebral activity at a limited anatomical range, while FC represents the function of blood oxygen signals between brain regions that are far away from each other at the network aspect. Therefore, the two analyses of ReHo and FC are credited with complementary and can jointly detect the synchronization of local and remote brain activity.^41^, ^42^ Therefore, we used the PFC as seed point to analyze the changes of brain FC in CUMS mice. It was found that the FC between the cerebral hemispheres corresponding to PrL and PrA in PFC of CUMS mice were significantly weakened, and the area of the connection area was reduced. It was consistent with the trend of ReHo in PFC of patients with clinical MDD and SVC monkeys.

Neuroinflammation caused by social pressure, mental factors, and various acute and chronic stress acts on a hinged role in the occurrence of depression. According to previous studies, inflammatory molecules such as IL‐6, C‐reactive protein, and IL‐1β in peripheral blood of patients with MDD have increased.^43^ However, the specific mechanism of inflammation activation is still unclear. The RAGE is a multiligand pattern recognition receptor involved in a variety of chronic inflammatory states and plays an important role in many diseases.^44^ RAGE can bind to AGEs, HMGB1, S100s, amyloid β‐protein, and other ligands. These ligands are some endogenous factors, collectively known as DAMPs, which are closely related to the occurrence of depression.^44^ RAGE exists on the cell membrane, which can induce neuronal stress injury and microglia activation, participate in oxidative stress, immune activation, aging and so on.^16^, ^44^, ^45^ The results showed that although there was no significantly statistical difference in the level RAGE of serum between MDD patients and normal people, the expression of RAGE and HMGB1 mRNA in peripheral leukocytes were significantly increased, and S100β mRNA expression was significantly decreased in MDD patients. The relative expression of RAGE and HMGB1 mRNA were positively correlated with HAMD and SDS scores, and S100β mRNA was negatively correlated with HAMD and SDS scores. These results suggested that inflammatory proteins of RAGE‐DAMPs are closely related to the occurrence of depression, which is consistent with previous reports. At the same time, compared with CON monkeys, ELISA showed that RAGE was upregulated in serum of SVC monkeys. The results of qPCR suggested that RAGE mRNA expression was increased in the mPFC of SVC monkeys. WB and IF detection showed that the protein expression of RAGE and HMGB1 were upregulated and S100β expression was downregulated in the mPFC of SVC monkeys. The expression of NF‐κB was increased in mPFC. Similar results were obtained in CUMS mice. Therefore, we have reason to think that the high expression of RAGE in PFC may be an important reason for depression.

To further verify our hypothesis, we designed experiments using RAGE*^–/–^* mice and RAGE inhibitor (FPS‐ZM1) and overexpression of RAGE in PFC. Interestingly, we found that there were no significant difference in body weight, level of BDNF in serum, behavioral tests, and functional connectivity of PFC between RAGE*^–/–^* mice and wild‐type mice, The results suggested that the absence of RAGE did not affect the normal life state, behavioral performance, serum BDNF level and functional connectivity of PFC. It is consistent with the reported effect of RAGE knockout on mice. At the same time, we found that RAGE*^–/–^* and intraperitoneal injection of FPS‐ZM1 could significantly reduce the weight loss, sugar consumption, and resting time of TST and FST and increased the level of BDNF in serum and downregulated the expression of NF‐κB, RAGE, and HMGB1 of PFC. It is suggested that RAGE knockout or inhibition can improve the depressive‐like behavior of mice, resist chronic stress, and inhibit the production of inflammatory proteins.

Furthermore, we overexpressed RAGE adeno‐associated virus (AAV) in PFC of wild‐type mice. We found that the consumption of sucrose was reduced, the resting time of TST and FST was significantly prolonged, the level of BDNF in serum was decreased, and the expression of NF‐κB, RAGE, and HMGB1 of PFC in mice was increased. These findings suggest that AAV9*^RAGE^* overexpression in PFC can induce depressive‐like behavior in mice, which complements our previous experimental results in depressed monkeys and mice. In addition, we found that lack of RAGE could increase the intensity of FC of prefrontal cortex (PrL and FrA) in mice after CUMS exposure, and the area of FC increased. Furthermore, RAGE plays an important role in the development of depression in mice. The absence of RAGE can improve the FC of PFC of mice under chronic stress, thus reducing the occurrence of depressive‐like behavior. Therefore, our results from three species level explain that chronic stress can induce the immune activation of RAGE‐DAMPs, which further leads to low functional state, weakened FC of PFC, and depressive‐like behavior.

The advantage of this study is to explore the mechanism of RAGE inPFC of depression by combining the complete set of human data (blood samples, functional magnetic resonance imaging, clinical data) collected by highly selected human single center, nonhuman primate, and rodent depression models. However, it is worth noting that the sample size is relatively small, so future research still needs a larger sample size to consolidate the current conclusion. Second, there is a lack of FC analysis between humans and primates. The improvement of data helps to better clarify the mechanism of depression and is highly encouraged. Next limitation is that the relationship between RAGE and other brain regions has not been deeply studied. The mechanism of brain network will be clarified in future work. Finally, for the animal (monkeys and mice) model, we have only used one of many stress depression models. In future studies, we will use other animal stress models to verify and strengthen our conclusion.

## 5 CONCLUSION

To sum up, this study unveiled the chronic stress can induce the inflammation and immune activation of RAGE‐DAMPs, resulting in brain dysfunction and weakening of FC of PFC, and depressive‐like behavior. The knockout or inhibition of RAGE can resist the effects of chronic stress on susceptibility, brain function, and behavior of depression. It further confirmed the important role of PFC in regulating emotional disorder, which provided molecular imaging basis for potential treatment strategies of depression.

## CONFLICT OF INTEREST

The authors declare no biomedical financial interests or potential conflicts of interest.

## AUTHOR CONTRIBUTIONS

YMB, TTG, and TZ collected clinical specimens and rs‐fMRI data, LPX verified human specimens, and YQL analyzed clinical data and rs‐fMRI data. WXY and DZ designed and carried out experiments on cynomolgus monkeys and mice, sorted out the data, and wrote the manuscript. XGS and YFS designed clinical experiments and guided animal experiments. ZYD revised the manuscript and GW supervised the clinical, monkey imaging parameters and quality. ZPL and LG supervised and designed the whole experiments and revised the manuscript. All authors contributed to experimental implementation and results interpretation, read, and approved the final manuscript.

## Supporting information

Supporting Information
